The article "Analysis of a five year experience of permanent pacemaker implantation at a Nigerian Teaching Hospital: need for a national database" was published in 2013. Journal: Pan Afr Med J.

# Analysis of a five year experience of permanent pacemaker implantation at a Nigerian Teaching Hospital: need for a national database

**DOI:** 10.11604/pamj.2013.16.16.2644

**Published:** 2013-09-15

**Authors:** Bode Falase, Michael Sanusi, Adeyemi Johnson, Fola Akinrinlola, Reina Ajayi, David Oke

**Affiliations:** 1 Cardiothoracic Division, Department of Surgery, Lagos State University College of Medicine, Lagos State University Teaching Hospital, Ikeja, Lagos, Nigeria; 2 First Cardiology Consultants, Ikoyi, Lagos, Nigeria; 3 Cardiology Unit, Department of Medicine, Lagos State University Teaching Hospital, Ikeja, Lagos, Nigeria

**Keywords:** Pacemaker, database, implantation, follow up, Nigeria

## Abstract

**Introduction:**

Permanent pacemaker implantation is available in Nigeria. There is however no national registry or framework for pacemaker data collection. A pacemaker database has been developed in our institution and the results are analyzed in this study.

**Methods:**

The study period was between January 2008 and December 2012. Patient data was extracted from a prospectively maintained database which was designed to include the fields of the European pacemaker patient identification code.

**Results:**

Of the 51 pacemaker implants done, there were 29 males (56.9%) and 22 females (43.1%). Mean age was 68.2±12.7 years. Clinical indications were syncopal attacks in 25 patients (49%), dizzy spells in 15 patients (29.4%), bradycardia with no symptoms in 10 patients (17.7%) and dyspnoea in 2 patients (3.9%). The ECG diagnosis was complete heart block in 27 patients (53%), second degree heart block in 19 patients (37.2%) and sick sinus syndrome with bradycardia in 5 patients (9.8%). Pacemaker modes used were ventricular pacing in 29 patients (56.9%) and dual chamber pacing in 22 patients (43.1%). Files have been closed in 20 patients (39.2%) and 31 patients (60.8%) are still being followed up with median follow up of 26 months, median of 5 visits and 282 pacemaker checks done. Complications seen during follow up were 3 lead displacements (5.9%), 3 pacemaker infections (5.9%), 2 pacemaker pocket erosions (3.9%), and 1 pacemaker related death (2%). There were 5 non-pacemaker related deaths (9.8%).

**Conclusion:**

Pacemaker data has been maintained for 5 years. We urge other implanting institutions in Nigeria to maintain similar databases and work towards establishment of a national pacemaker registry.

## Introduction

Bradyarrhythmias are a cause of sudden death in Nigeria, though the precise incidence is unknown. Pacemaker implantation is an accepted intervention which has been shown to improve the quality of life and reduce mortality in patients with bradyarrhythmias. Published experience in Nigeria has shown that implantation rates are low, the main indication for implantation is complete heart block (CHB) and most patients receive ventricular implants [1]. Pacemaker implantation is however not widely available, is difficult for the average Nigerian to access, and when available is often expensive [2]. Few institutions in Nigeria therefore offer pacemaker implantation or follow up services. It is of concern that the few implantations being performed are often not formally documented as there is currently no national framework for pacemaker data collection.

The article "Analysis of a five year experience of permanent pacemaker implantation at a Nigerian Teaching Hospital: need for a national database" was published in 2013. Journal: Pan Afr Med J.

A pacemaker implantation and follow up service was established in our institution in 2008. The aim of this study was to review our experience by analysis of our pacemaker database.

## Methods

### Institutional Settings

Following patient referral the clinical indication for pacemaker therapy is established from the history and the diagnosis confirmed with a 12 lead ECG (and 24 hour holter if necessary). Cardiac function is assessed with a transthoracic echocardiogram. Pacemaker implantation is performed in a dedicated theatre suite equipped with a fluoroscopic C arm. The implantation team is composed of a surgeon who performs the implantation, a cardiac physiologist who performs the checks of pacemaker parameters, a pacemaker technician to operate the fluoroscope for imaging and a scrub nurse. Monitored parameters are the heart rhythm, heart rate, non-invasive blood pressure and peripheral oxygen saturation. A standard subclavian approach is used after infiltration with local anaesthesia in all cases. Prior to lead fixation the R wave (P wave if atrial lead) and pacing threshold are checked. Target values are R wave greater than 6 millivolts (mV), P wave greater than 2 mV, lead impedance less than 1200 Ohms and pacing threshold less than 1 volt (V). Diaphragmatic pacing is checked at 10V. The pacemaker pocket is irrigated with 1g of ceftriaxone, the pacemaker lead connected to the pulse generator and the wound closed in layers. An arm sling is used in all cases to restrict movement of the arm on the operation side (to reduce the risk of lead displacement) and the patient is transferred to the ward.

Patients are monitored on the ward for 48 hours to exclude lead displacement. After 48 hours a pacemaker check is done and the patient is given a copy of both the pacemaker implantation report (Figure 1) and pacemaker check report (Figure 2) prior to discharge. Patients are counseled to maintain the arm sling for a week and return for pacemaker checks. Pacemaker check sequence is 6 weeks, 3 months, and then every 4 months for a year. After a year the checks are done every 6 months. Pacemaker checks are performed mainly by the cardiac physiologists and complications reported to the surgeon. A pacemaker check report is generated after each visit, and a copy is given to the patient and a copy kept on file. Contact details of all patients are maintained on the database so that contact can be made if any appointment is missed.

The article "Analysis of a five year experience of permanent pacemaker implantation at a Nigerian Teaching Hospital: need for a national database" was published in 2013. Journal: Pan Afr Med J.

**Figure 1:** Sample pacemaker implant report

**Figure 2:** Sample pacemaker check report

### Patient Data

A Microsoft Access database was designed and has been maintained prospectively since the inception of the programme in January 2008. Data storage covers the fields recommended by the European pacemaker patient identification codes [3]. Sample snapshots from the database are shown in Figure 3, Figure 4. Permission was obtained from the Ethics committee of the Lagos State University Teaching Hospital for use of the existing patient data from the database. For the purpose of this study the records of all implants between January 2008 and December 2012 were extracted for analysis. The records analyzed were those of the 51 patients that had been implanted in our institution, excluding 7 patients referred for follow up who had not been implanted in our institution. Data fields selected for analysis were patient demographics, clinical indications for pacemaker therapy, electrocardiographic diagnosis, distribution of pacemakers by manufacturer, distribution by pacemaker mode, distribution by implantation year, completeness of follow up and complications noted on follow up. Data analysis was done with Microsoft Excel 2010. The results are presented as numbers and percentages as appropriate. Summary data is presented as mean±standard deviation.

**Figure 3:** Snapshot of pacemaker database showing Pacemaker implant form

**Figure 4:** Snapshot of pacemaker database shower pacemaker check form

## Results

Of the 51 patients implanted there were 29 males (56.9%) and 22 females (43.1%). Ages ranged from 22-92 years with a mean age of 68.2±12.7 years. Age distribution is as shown in Figure 5.

**Figure 5:** Distribution in percentages of implants by patient age and decade of life

The distribution of clinical indications for pacemaker therapy was syncopal attacks in 25 patients (49%), dizzy spells in 15 patients (29.4%), documented bradycardia with no symptoms in 10 patients (17.7%) and dyspnoea/heart failure in 2 patients (3.9%). The ECG diagnosis was Complete Heart Block (CHB) in 27 patients (53%), second degree heart block (SDHB) in 19 patients (27.2%) and Sick Sinus Syndrome with bradycardia (SSS) in 5 patients (9.8%). There was no patient with atrial fibrillation.

The article "Analysis of a five year experience of permanent pacemaker implantation at a Nigerian Teaching Hospital: need for a national database" was published in 2013. Journal: Pan Afr Med J.

The distribution by pacemaker manufacturer was Medtronic (Minneapolis Minnesota USA) in 33 patients (66.7%), Pacetronix (Kolkata India) in 10 patients (19.6%) and St Jude (St Paul Minnesota USA) in 7 patients (13.7%). Pacing modes used were VVI (Ventricular Demand Pacing) in 9 patients (17.6%), VVIR (Rate Responsive Ventricular Demand Pacing) in 20 patients (39.2%), DDD (Dual Chamber Demand Pacing) in 2 patients (3.9%) and DDDR (Rate Responsive Dual Chamber Demand Pacing) in 20 patients (39.2%). Overall single chamber ventricular pacing (VVI(R)) was used in 29 patients (56.9%) and dual chamber pacing (DDD(R)) in 22 patients (43.1%) with a progressive annual reduction in the use of ventricular pacing and an increased use of dual chamber pacing over the study period (Figure 6). Distribution of implant mode by diagnosis is shown in Table 1. Of the 51 ventricular leads, active fixation leads were used in 29 patients (56.9%) and passive fixation in 22 patients (43.1%). Atrial pacemaker leads were active fixation in all 22 patients with dual chamber systems. A temporary pacemaker was used in only 1 patient. The cephalic vein was never used for venous access, access being the left subclavian vein in 35 patients (68.6%) and the right subclavian vein in 16 patients (31.4%).

**Figure 6:** Distribution of implants by mode and year

**Table 1:** Distribution of Implants by diagnosis and mode

Diagnosis	VVI	VVIR	DDD	DDDR	Total
2nd Degree HB-Wenckebach			1	1	2
2nd Degree HB-Mobitz	2	7		8	17
CHB	7	12		8	27
SSS		1	1	3	5
**Total**	9	20	2	20	51

CHB: Complete Heart Block, SSS: Sick Sinus Syndrome; VVI: Ventricular Demand Pacing; VVIR: Rate Responsive Ventricular Demand Pacing; DDD: Dual Chamber Demand Pacing; DDDR: Rate Responsive Dual Chamber Demand Pacing)

At implantation the average R wave obtained was 11.8±4.6 mV while the average P wave obtained was 2.9 + 1.8 mV. The average atrial pacing threshold was 0.65±0.54 V and the average ventricular pacing threshold was 0.59±0.39 V. Average impedance for the atrial leads was 650.2±191.7 Ohms and was 780.5±230.2 Ohms for the ventricular leads. Complications seen postoperatively and during follow up were 3 lead displacements (5.9%), 3 pacemaker infections (5.9%), 2 pacemaker pocket erosions (3.9%), and 1 pacemaker related death (2%). Details of complications seen and time interval from implantation when they occurred are shown in Table 2.

**Table 2:** Complications seen during follow up and outcomes

Implant Number	Sex	Age	Mode	Complication	Interval	Outcome
**7**	Male	81	VVI	Pacemaker pocket erosion	3 years	Removal of pulse generator and VVIR implant opposite side
**8**	Female	79	DDD	Ventricular lead exit block	2 years	Refused re-implant. Sudden death
**9**	Male	67	DDDR	Atrial lead displacement	3 days	Refused reoperation. Mode changed to VVIR
**10**	Female	71	VVIR	Pulse generator migration, lead displacement	4 years	Removal of pacing system. New DDDR implant opposite side
**11**	Male		DDDR	Myocardial infarction	48 hours	Non pacemaker related death
**21**	Male	29	VVIR	Pacemaker pocket erosion	3 years	Removal of pulse generator and DDDR implant opposite side
**22**	Female	72	VVIR	Lead displacement	24 hours	Lead repositioned
**37**	Male	60	DDDR	Pacemaker pocket infection	2 weeks	Removal of pacing system. New DDDR implant opposite side
**45**	Male	69	DDDR	Pacemaker pocket infection	3 weeks	Removal of pacing system. New DDDR implant opposite side
**49**	Female	72	DDDR	Pacemaker pocket infection	4 days	Removal of pacing system. New DDDR implant opposite side

VVI: Ventricular Demand Pacing, VVIR: Rate Responsive Ventricular Demand Pacing; DDD: Dual Chamber Demand Pacing, DDDR: Rate Responsive Dual Chamber Demand Pacing

At follow up in the pacemaker clinic, 282 pacemaker checks have been done on the 51 patients implanted in our institution. Of these 51 patients, 31 patients (60.8%) still remain under follow up in the pacemaker clinic. For these patients, the follow up period has ranged from 1-60 months with a median follow up of 26 months. The number of clinic visits ranged from 114 with a median of 5 visits.

The article "Analysis of a five year experience of permanent pacemaker implantation at a Nigerian Teaching Hospital: need for a national database" was published in 2013. Journal: Pan Afr Med J.

File closure has been done in 20 patients (39.2%). The reasons for file closure were pacemaker removal in 5 patients (25%), non-pacemaker related death in 5 patients (25%), transfer to another hospital in 5 patients (25%), lost to follow up in 2 patients (10%), inability to attend from transportation problems in 2 patients (10%) and pacemaker related death in 1 patient (5%). Of the 5 non-pacemaker related deaths, 4 patients were reported to have suffered myocardial infarctions while 1 patient died of complications of prostate cancer.

## Discussion

There are currently 10 centres in Nigeria known to implant pacemakers. There are 3 centres in Lagos and 1 each in Enugu, Ibadan, Abuja, Port Harcourt, Calabar, Ife and Ilorin (personal data). To date a centre in Lagos [1] and the centre in Enugu [4] have published their experience. In the experience of Thomas et al from Lagos, 100 patients were implanted between 1999 and 2004. Average age was 62 years, 93% of patients were female, 86% of patients were diagnosed with CHB and overall 89% received single chamber ventricular pacing and 11% received dual chamber pacing,. No complications were recorded [1]. The Enugu experience is a smaller series of 23 implants done between 2001 and 2006 in which the mean age was 70 years, 65% of patients were in CHB, endocardial leads were used in 65% of cases, and epicardial leads in 35% of cases [4]. There is also published experience in 2003 from Dakar Senegal of 92 implants over a 3 year period. There was an equal male to female ratio and 87% of implants were single chamber ventricular pacing. Interestingly 53% of the pacemakers implanted were donated recycled pacemakers. Complications seen in the series were pacemaker infections in 5 patients, 3 lead displacements, 1 pacemaker syndrome and 8 patients that died during follow up of non-pacemaker related causes [5].

The article "Analysis of a five year experience of permanent pacemaker implantation at a Nigerian Teaching Hospital: need for a national database" was published in 2013. Journal: Pan Afr Med J.

The mean age in our series was 68 years with 56.9% being male and 43.1% female. This is within the mean age range of 65 to 75 years reported in the 11^th^ World survey of cardiac pacing and implantable cardioverter-defibrillators [6]. Additionally the 11^th^ world survey showed that there are slightly more males receiving implants than females (about 55% male, 45 % females) which is similar to our experience. The use of dual chamber pacing in 43.1% of patients in our series is considerably higher than reported in other West African series and reflects the worldwide trend of increased use of dual chamber pacing seen in the 11^th^th World survey. Similar to the findings of other West African series, most patients in our environment are diagnosed with CHB and about 50% present having had syncopal attacks. This is unlike the pattern in the Western World where 30% or less of patient present with CHB and Sinus Node Dysfunction (SND) is the predominant indication for cardiac pacing [6].

Maintaining a stock of pacemakers locally makes it easier to proceed directly to permanent pacemaker implantation. In this series of 51 patients, only one temporary pacemaker was implanted. This is unlike the earlier experience from Lagos [1] where 6 patients required temporary pacing as a bridge to permanent pacemaker implantation due to delays in procuring the pacemaker. At the period of that publication pacemaker implantation services were still being developed. In the ensuing 5 years since that publication some progress has been made and some pacemaker manufacturers now have local representation in Nigeria, enabling purchase of pacemakers locally as opposed to waiting weeks for importation. It has been recommended that it is unnecessary to implant a temporary pacemaker if there is immediate access to a permanent pacemaker [7] and this is our current practice.

In our practice there has been a progressive decrease in the use of single chamber ventricular pacing and an increase in dual chamber pacing over the last 5 years of our experience. In the 1990s initial recommendations urged more use of dual chamber pacing as it was thought that the hemodynamic benefits of AV synchrony would translate into improved longevity, improved quality of life and reduction in strokes [8]. The first randomized controlled trial by Andersen et al (AAI vs. VVI) showed reduced mortality and improved quality of life as advantages of atrial based pacing (or dual chamber pacing) over ventricular based pacing [9, 10]. However 3 subsequent large prospective randomized controlled trials reported between 2000 and 2002 contradicted these findings. These were MOST (DDDR vs. VVIR) [11], CTOPP (DDD(R) vs. AAI(R) or VVI(R)) [12] and UKPACE (DDD vs. VVI(R)) [13]. (MOST: Mode Selection Trial, CTOPP: Canadian Trial of Physiological Pacing, UKPACE: The United Kingdom Pacing and Cardiovascular Events Trial). These trials showed that overall mortality, cardiovascular events, strokes, hospital admission for heart failure and the development of pacemaker syndrome (apart from in the MOST trial) were similar for atrial based pacing (AAI(R)/ DDD(R)) and ventricular pacing (VVI(R)/DDD(R)). The main benefit of atrial based pacing appeared to be a risk reduction in the development of chronic atrial fibrillation. This risk reduction applied to patients who had pacemakers implanted for high Atrio-ventricular block (AVB) in the UKPACE trial, SND (Sinus Node Disease) in the MOST trial, SND and AVB in the CTOPP trial. It has been suggested that the evidence now shows that the guidelines should be changed to reflect the fact that atrial based pacing (dual chamber pacing) is not recommended over ventricular pacing to improve survival or stroke [14]. However despite the results of these trials, recommendations have not changed and dual chamber pacing still predominates in the Western World. How do these findings apply to West African patients? The patient population is different as unlike the Western series where SND is the main indication for cardiac pacing West African experience confirms AVB as the main indication in this region. Only the UKPACE trial specifically addressed cardiac pacing in patients over 70 with AVB. Whether these findings can be extrapolated to the West African population is unknown.

The article "Analysis of a five year experience of permanent pacemaker implantation at a Nigerian Teaching Hospital: need for a national database" was published in 2013. Journal: Pan Afr Med J.

It has been suggested that dual chamber pacing though more expensive may be offset by reduced replacement for pacemaker syndrome and improved quality of life [15]. None of the patients in our series developed pacemaker syndrome, despite 56.8% of implants being single chamber ventricular implants. 89% of the patients in the series by Thomas et al received ventricular implants with no report of pacemaker syndrome [1] which is similar to the experience from Senegal where 87% of patients had ventricular implants and only 1 pacemaker syndrome was reported [4]. The increased use of ventricular pacing in West Africa is driven largely by cost as cardiac pacing is not covered by insurance and is largely self funded [2]. Since ventricular pacing appears to be well tolerated and is cheaper, should this be the preferred option for our patients? Complication rates seen in this study are comparable to other West African series. The major complications of pacemaker pocket infection in 3 patients (5.9%) and lead displacement in 3 patients (5.9%) compares favorably with the experience from Senegal where the pacemaker infection rate was 5.4% of patients [5]. This is however higher than the 1.5% pacemaker infection rate in a series of 1,286 implants in the UK reported recently [7]. Of note is the fact that every patient implanted in our series is followed up closely, enabling complications to be promptly addressed (Table 2). Our detailed follow up may account for a higher pick up rate of complications, in contrast to the earlier reported experience of Thomas et al where no complications were noted in 100 implants over a five year period [1].

We noted that all the pacemaker infections occurred in dual chamber implants. It has been shown that there can be a higher complication rate with dual chamber implants [13]. We will monitor this closely as if this trend persists it could be a further deterrent to using dual chamber implants as it puts more of a financial burden on the patient and relations who would need to raise further funds for a second implant.

We have considered the re-use of pacemakers as there is some evidence that it is safe and could reduce costs for patients [16]. Average implantation rates in our series was 10 implants per year, whereas in the Senegal experience the implant rate was as high as 30 implants a year, due to the high use of donated recycled pacemakers [5]. This may be an option worth considering unless pacemaker manufacturers can substantially reduce the cost of pacemakers in Nigeria to make this life saving intervention more accessible.

Only 1 pacemaker related death occurred in this series. This occurred in an elderly patient who received a Pacetronix implant (VVI) with a tined, non-steroid eluting endocardial lead. Over a period of 2 years there was a gradual rise in pacing threshold from implantation level of 0.8V to 2.5V. Pacing amplitude had been increased to 5V and the patient advised on a change of implant. She however declined and died suddenly, presumably from sudden failure to capture. This singular experience informed our current practice where we no longer use Pacetronix implants and all pacemaker leads used are steroid eluting and active fixation.

The article "Analysis of a five year experience of permanent pacemaker implantation at a Nigerian Teaching Hospital: need for a national database" was published in 2013. Journal: Pan Afr Med J.

Of the 5 non-pacemaker related deaths, 4 were reported as being secondary to myocardial infarctions. Diagnosis of myocardial infarction was made by cardiac enzymes and electrocardiogram changes in 1 patient, and purely from ECG changes in the other 3 patients. The incidence of Ischaemic heart disease (IHD) is known to be on the increase in Nigeria [17] so the co-existence of IHD and bradycardia needs to be considered in elderly patients presenting for pacemaker therapy.

There is great variability in implantation rates between different countries as shown in the 11th World survey of cardiac pacing and implantable cardioverter-defibrillators [6]. The largest implanting nation was the USA with 235,567 new implants. Other high implanters were Germany (76,046), France (48,487), Italy (44,653), Japan (34,813) and India (20,000). The number of centres per country varied with the USA having 3,400 implanting centres, Japan 2,300 centres, India 738 centres, China 783 centres, Germany 986 centres, France 550 centres and the UK 211 centres. 30-150 implants were done in each centre. Africa and the Middle East made up one group of seven countries in this report and the number of implanting centres in this group was Iran 54, South Africa 49, Israel 20, Sudan 4, and Bahrain Oman and Qatar with 1 centre each. The annual number of implants in these centres was Iran 3,373, Israel 3,000, South Africa 2,939, Sudan 180, Oman 92, Qatar 57 and Bahrain 48.

In the midst of this great variability in the number of pacing centres and implants done per country, it is of great concern that Nigeria was not included in this survey. This stresses the urgency in establishment of a framework for a national registry so that the efforts of various implanting institutions in Nigeria can be captured.

## Conclusion

A pacemaker implantation and follow up service has been established in our institution and a robust database has been developed and maintained. Early results show that the main indications for implantation are complete heart block and second degree heart block. Use of dual chamber pacing is higher than has been reported from other West African Centres. Continued patient follow up may be able to address questions of pacemaker therapy unique to our environment. Complications rates have been low. Complete follow up information is available for 49 patients (96%). We urge other implanting institutions in Nigeria to maintain similar databases and work towards establishment of a national pacemaker registry.
